The article "Blind Image Inpainting with Mixture Noise Using ℓ0 and Total Regularization" was published in 2022. Journal: Comput Math Methods Med.

# Blind Image Inpainting with Mixture Noise Using *ℓ*_0_ and Total Regularization

**DOI:** 10.1155/2022/3180612

**Published:** 2022-09-30

**Authors:** Xiaowei Xu, Shiqi Geng

**Affiliations:** College of Physics and Electronic Electrical Engineering, Huaiyin Normal University, Huaian, China

## Abstract

The blind image inpainting problem need to be handle when faced with a large number of images, especially medical images in medical health. For the proposed nonconvex sparse optimization model, a proximal based alternating direction method of multipliers (PADMM) method is designed to solve the problem. Firstly, *ℓ*_0_ sparse regularization is imposed to the binary mask since the missing pixels are sparse in our experiments. Secondly, the total variation term is utilized to describe the underlying clean image. Finally, *ℓ*_2_ regularization of the fidelity term is used to solve the given blind inpainting problem. Experiments show that this method has better performance than traditional method, and could deal with the blind image inpainting problem.

## 1. Introduction

Medical images can directly reflect the function and health status of human tissues, and have become one of the standards of diagnosis and medical intervention. With the increasing availability and utilization of modern medical imaging such as disease database, X-ray film and magnetic resonance imaging, the demand for automatic processing of medical image data is increasing. With the application of medical images, automatic medical image analysis has become one of the hot directions of contemporary medical imaging research [1, 2]. In the process of image capture, imaging sensors broken or the error in information transmission may cause some pixels missing or corrupted by impulse noise [3–8].

In this work, the image is defined as a vector with *n* pixels in lexicographic ordering, *x* ∈ *ℜ*^*n*^. It can be represented mathematically as follows:

(1) $$\begin{array}{c} y=Ax \end{array}$$

where *y* ∈ *ℜ*^*n*^ is the observed image, *x* ∈ *ℜ*^*n*^ is the clean image and *A* ∈ *ℜ*^*n*×*n*^ is an identity matrix. If the clean image *x* is corrupted by the additive Gaussian noise *η*_*g*_, the model will be updated as follows:

(2) $$\begin{array}{c} y=A\left(x+\eta_{g}\right) \end{array}$$

The image is corrupted by impulse noise, and the pixels in *y* is corrupted by the impulse noise *η*_*i*_. The blind image inpainting model with the mixture noise (Gaussian and impulse noise) is finally described as follows [9]:

(3) $$\begin{array}{c} y=A\left(x+\eta_{g}\right)+\left(I_{n}-A\right)\eta_{i} \end{array}$$

How to solve the E.q. (2) efficiently and effectively is the most important issue. It is clear that E.q. (2) is quite challenging. It has three unknown term *A*, *η*_*g*_ and *η*_*i*_. The goal of this paper is to estimate the clean image *x* from the partial observation *y* without unknow mask *A,* noise *η*_*g*_ and *η*_*i*_.

The article "Blind Image Inpainting with Mixture Noise Using ℓ0 and Total Regularization" was published in 2022. Journal: Comput Math Methods Med.

In the earlier researches, the inpainting problem can be solved by many approaches related image reconstruction from the aspect of sparse modeling [10–13]. More common strategies for the removal of impulse noise for blind inpainting problems are to estimate an approximated A by computing the support set of the noisy pixels with some outlier detection methods, and apply the reconstruction methods for a known mask A.

The difficulty of reconstructing an image with missing data and mixture noise is basically to detect the locations of outliers. Some filtering based methods estimate the missing values, such as the adaptive median filter [14], and adaptive center weighted median filter [15].

Two phase based methods for blind inpainting problems involve the estimation of mask A, which is calculated by some outlier detection approaches. After the mask estimation, the inpainted image is generated by the image reconstruction step, which is implemented by a standard convex optimization. Some convex methods were ulitized to estimate the inpainted images [16]. Used the total variation (TV) regularizer [17] estimates the inpainted images. Xiao et al. [18] proposed a combination of *ℓ*_1_-norm and *ℓ*_0_-norm regularizers for simultaneously removing impulse noise and computing learning dictionary after the mask. In addition, the authors [19] presented an approach for mixed impulse and Gaussian noise removal. In the approach, a logarithmic transformation strategy is applied to convert the multiplication between the image and binary mask. Then, the image and mask terms are estimated iteratively with TV regularization applied on the image. Especially, the method can also be extended to the removal of impulse noise by relaxing the regularizer from the *ℓ*_0_ norm to the *ℓ*_1_ norm.

Some approaches could estimate the mask and impulse noise field by an iterative process instead of involving a separated mask detection step, such as a low-rank matrix recovery method [20]. The proposed approach belongs to the category of simultaneously estimating the mask and impulse noise.

To address the challenging blind inpainting task with mixture noise, a novel model is proposed based on imposing a *ℓ*_0_ sparse regularization to the binary mask. The proposed model can be efficiently solved by a designed proximal based alternating direction method of multipliers (PADMM) method. The main contribution of this work is given as follows: 1) A new model that fits in the practical situation of blind inpainting problem is proposed. 2) The new model solves the challenging blind inpainting task with mixture noise. 3) An efficient algorithm is given to effectively solve the proposed model.

The article "Blind Image Inpainting with Mixture Noise Using ℓ0 and Total Regularization" was published in 2022. Journal: Comput Math Methods Med.

The outline of this paper is given as follows. The proposed method including the new model and the designed algorithm is exhibited in Section 2. The solution of the proposed method is described in Section 3.  Section 4 shows the experimental results and analysis. Finally, we draw some conclusions in Section 5.

## 2. Model Building

The paper proposes a minimization model to solve the image inpainting problem on the basic blind image with mixture noise. we denote a as the verctor form of mask A and the E.q. (3) can be expressed as follows:

(4) $$\begin{array}{c} y=a⊗\left(x+\eta_{g}\right)+\left(Ι-a\right)⊗\eta_{i} \end{array}$$

where ⊗ stands for a dot product between vectors, and *Ι* is a vector with all the value *Ι*.

*x* ∈ *ℜ*^*n*^ is the vector form of one matrix *x* ∈ *ℜ*^*n*1×*n*2^ with *n* = *n*1 × *n*2 in (2), and *a*, *y* are the vectors with the same dimensions as *x*. As a is the position of pixels missing, the *Ι*-*a* represents the locations of impulse noise in the image.

we will give more explanations for E.q.(4) to present the proposed model for the blind image inpainting with mixture noise:

Since *a* ⊗ (*y* − *x*) mainly represents Gaussian noise, we use the *ℓ*_2_ norm ‖*a* ⊗ (*y* − *x*)‖_2_^2^ to construct the fidelity term^3^
2. (1‐*a*) ⊗ *y* only represents impulse noise (e.g., salt-peppers, random value), thus we may use *ℓ*_1_ sparse regularization to describe (1‐*a*) ⊗ *y*, *i*.*e*., ‖(1‐*a*) ⊗ *y*‖_1_
Especially, if the impulse noise is relatively dense, it may impose £q regularization to a in the new model, i.e., ‖*a*‖_0_. Otherwise, if the impulse noise is sparse and the condition of minimizing ‖*a*‖_0_ may not hold, we could easily set a small parameter to control it
Finally, we employ the (anisotropic) total variation (TV) regularization to the underlying clean image x, i.e., ‖∇*x*‖_1_, the TV regularization is quite popular and useful in the applications of image processing

As presented above, we formulate the final proposed model for the inpainting task as follows:

(5) $$\begin{array}{c} \left(x,a\right)=\arg\underset{x,a}{\min}\frac{1}{2}{\left\|a⊗\left(y-x\right)\right\|}_{2}^{2}+\lambda_{1}{\left\|\nabla x\right\|}_{1}+\lambda_{2}{\left\|a\right\|}_{0}+\lambda_{3}{\left\|\left(1-a\right)⊗y\right\|}_{1} \end{array}$$

The *ℓ*_0_ minimization $\underset{a}{\min}{\left\|a\right\|}_{0}$ can be equality described as $\underset{v}{\min}<1,1-v>$ such that *v* ⊗ |*a*| = 0 and 0 ≤ *v* ≤ 1 based on [8]. Thus, E.q.(2) can be expressed as follows:

(6) $$\begin{array}{c} \begin{array}{c} \underset{x,a,z,w,v}{\min}\frac{1}{2}{\left\|a⊗\left(y-x\right)\right\|}_{2}^{2}+\lambda_{1}{\left\|z\right\|}_{p,1}+\lambda_{2}<1,1-v>+\lambda_{3}{\left\|w\right\|}_{1}\\ s.t.\nabla x=z,v⊗\left|a\right|=0,0\leq v\leq 1,\left(1-a\right)⊗y=w \end{array} \end{array}$$

As discussed above, we may get the following augmented Lagrangian problem instead of the constrained minimization E.q. (6) with variable substitution.

(7) $$\begin{array}{c} \begin{array}{c} \zeta \left(x,a,z,w,v,\pi_{1},\pi_{2},\pi_{3}\right)=\frac{1}{2}{\left\|a⊗\left(y-x\right)\right\|}_{2}^{2}+\lambda_{1}{\left\|z\right\|}_{p,1}+\lambda_{2}<1,1-v>+\lambda_{3}{\left\|w\right\|}_{1}+<\pi_{1},\nabla u-z>+\frac{\beta_{1}}{2}{\left\|\nabla u-z\right\|}_{2}^{2}+<\pi_{2},v⊗\left|a\right|>+\frac{\beta_{2}}{2}{\left\|v⊗\left|a\right|\right\|}_{2}^{2}+<\pi_{3},\left(1-a\right)⊗y-w>+\frac{\beta_{3}}{2}{\left\|\left(1-a\right)⊗y-w\right\|}_{2}^{2}\\ s.t.0\leq v\leq 1 \end{array} \end{array}$$

Where *π*_1_, *π*_2_ and *π*_3_ are Lagrange multipliers, and *β*_1_, *β*_2_ and *β*_3_ are three positive parameters. The Lagrangian problem *ζ*(*x*, *a*, *z*, *w*, *v*, *π*_1_, *π*_2_, *π*_3_) can be solved alternatively and iteratively by the following minimization subproblems in Section 3.

The article "Blind Image Inpainting with Mixture Noise Using ℓ0 and Total Regularization" was published in 2022. Journal: Comput Math Methods Med.

## 3. Model Solution Method

We add the proximal term 1/2‖*x* − *x*^*k*^‖_*D*_^2^ to the x subproblem from E.q.(7) and denote ‖*x*‖_*D*_^2^ = *x*^*T*^*Dx* to get the following proximal

(8) $$\begin{array}{c} x^{k+1}=\arg\underset{x}{\min}\frac{1}{2}{\left\|a⊗\left(y-x\right)\right\|}_{2}^{2}+<\pi_{1},\nabla u-z>+\frac{\beta_{1}}{2}{\left\|\nabla u-z\right\|}_{2}^{2}+\frac{1}{2}{\left\|x-x^{k}\right\|}_{D}^{2} \end{array}$$

Where

(9) $$\begin{array}{c} D=\frac{1}{\kappa }{Ι}_{n}-\left(\mathrm{diag}\left(a\right)+\beta_{1}\nabla^{T}\nabla \right),\kappa \in \left(0,\left(\frac{1}{1+\beta_{1}{\left\|\nabla \right\|}^{2}}\right)\right) \end{array}$$

The solution of E.q.(8) is given as follows:

(10) $$\begin{array}{c} x^{k+1}=\frac{1}{2}{\left\|x-p^{k}\right\|}_{2}^{2} \end{array}$$

Where

(11) $$\begin{array}{c} p^{k}=x^{k}-\kappa_{1}\left[a⊗\left(x^{k}-y\right)+\nabla^{T}\left(\pi_{1}-\beta_{1}z\right)+\beta_{1}\nabla^{T}\nabla x^{k}\right] \end{array}$$

The *a*-subproblem is shown as the following:

(12) $$\begin{array}{c} a^{k+1}=\arg\underset{a}{\min}\frac{1}{2}{\left\|a⊗\left(y-x\right)\right\|}_{2}^{2}+<\pi_{2},v⊗\left|a\right|>+\frac{\beta_{1}}{2}{\left\|v⊗\left|a\right|\right\|}_{2}^{2}+<\pi_{3},\left(1-a\right)⊗y-w>+\frac{\beta_{3}}{2}{\left\|\left(1-a\right)⊗y-w\right\|}_{2}^{2} \end{array}$$

We need to discuss the solution by the following two cases:

When a >0,

(13) $$\begin{array}{c} a^{k+1}=\frac{-v⊗\pi_{2}+\beta_{3}y⊗Ι⊗y+y⊗\pi_{3}}{\left(y-x\right)⊗\left(y-x\right)+\beta_{2}v⊗v+\beta_{3}y⊗y} \end{array}$$

When a <0,

(14) $$\begin{array}{c} a^{k+1}=\frac{v⊗\pi_{2}+\beta_{3}y⊗Ι⊗y+y⊗\pi_{3}}{\left(y-x\right)⊗\left(y-x\right)+\beta_{2}v⊗v+\beta_{3}y⊗y} \end{array}$$

Therefore, the reformulation is:

(15) $$\begin{array}{c} y^{k+1}=\mathrm{sgn}\left(q^{k}\right)*\frac{{\left|q\right|}^{k}-v⊗\pi_{2}}{h^{k}} \end{array}$$

Where

(16) $$\begin{array}{c} q^{k}=\beta_{3}y⊗y+y⊗\pi_{3},h^{k}=\left(y-x\right)⊗\left(y-x\right)z+\beta_{2}v⊗v+\beta_{3}y⊗y \end{array}$$

The *z*-subproblem can be written as the following minimization problem:

(17) $$\begin{array}{c} z^{k+1}=\arg\underset{z}{\min}\lambda_{1}{\left\|z\right\|}_{1}+<\pi_{1},\nabla u-z>+\frac{\beta_{1}}{2}{\left\|\nabla u-z\right\|}_{2}^{2} \end{array}$$

which has a closed-form solution by soft-thresholding [7].

(18) $$\begin{array}{c} z^{k+1}=S\text{h}rink\left(\nabla x+\frac{\pi_{1}}{\beta_{1}},\frac{\lambda_{1}}{\beta_{1}}\right) \end{array}$$

Where

(19) $$\begin{array}{c} Shrink\left(x,t\right)=\max\left(0,\left|x\right|-\frac{1}{t}\right).*\mathrm{sign}\left(x\right) \end{array}$$

Similarly, the *w*-subproblem is given as the follows:

(20) $$\begin{array}{c} w^{k+1}=\arg\underset{w}{\min}\lambda_{3}{\left\|w\right\|}_{1}+<\pi_{3},\left(1-a\right)⊗y-w>+\frac{\beta_{3}}{2}{\left\|\left(1-a\right)⊗y-w\right\|}_{2}^{2} \end{array}$$

which holds the closed-form solution by soft-thresholding:

(21) $$\begin{array}{c} z^{k+1}=S\text{h}rink\left(\left(1-a\right)⊗y+\frac{\pi_{3}}{\beta_{3}},\frac{\lambda_{3}}{\beta_{3}}\right) \end{array}$$

The *v*-subproblem is given as the follows:

(22) $$\begin{array}{c} v^{k+1}=\arg\underset{0\leq v\leq 1}{\min}\lambda_{2}<1,1-v>+<\pi_{2},v⊗\left|a\right|>+\frac{\beta_{2}}{2}{\left\|v⊗\left|a\right|\right\|}_{2}^{2} \end{array}$$

which could also hold the closed-form solution [9]:

(23) $$\begin{array}{c} v^{k+1}=\min\left(1,\max\left(0,r^{k}\right)\right) \end{array}$$

Where

(24) $$\begin{array}{c} r^{k}=\frac{\lambda_{2}-\left|a\right|⊗\pi_{2}}{\beta_{2}\left|a\right|⊗\left|a\right|} \end{array}$$

We finally update the Lagrange multipliers by:

(25) $$\begin{array}{c} \pi_{1}^{k+1}=\pi_{1}^{k}+\beta_{1}\left(\nabla x^{k+1}-z^{k+1}\right),\pi_{2}^{k+1}=\pi_{2}^{k}+\beta_{2}\left(v⊗\left|a\right|\right),\pi_{3}^{k+1}=\pi_{3}^{k}+\beta_{3}\left(\left(1-a\right)⊗y-w\right) \end{array}$$

We may effectively obtain the solution of the constrained model (5) with the initial guesses *u*^0^ = *v*^0^ = *a*^0^ = 0. We summarize the above steps to get the following Algorithm 1:

Although Algorithm 1 involves some parameters, these parameters are actually not sensitive and easy to select. We also compute the energy of each iteration. If the energy is below a given tolerance, the iteration will stop and output the final result.

The article "Blind Image Inpainting with Mixture Noise Using ℓ0 and Total Regularization" was published in 2022. Journal: Comput Math Methods Med.

In the next section, we will exhibit the experiment results to demonstrate the effectiveness of the proposed method.

## 4. Experimental Results and Analysis

The numerical experiments in this section are implemented with MATLAB (R2016a) for both simulated and real images. The experimental computer has 2G RAM and Intel(R) Core(TM)i3-2370 M CPU: @2.40GHz 2.40GHz. Since the literatures for blind image inpainting with mixture noise are limited, we here only compare the proposed method with one recent state-of-the-art blind inpainting approach [6], denoted as “ASInpaint” ^4^.

In Figure 1, we present the whole process of image, which is degraded jointly by Gaussian noise and impulse noise. The goal of this work is to recover the clean image X from the degraded image Y. To evaluate the quantitative performance of the compared approaches, we employ two kinds of metrics to estimate the performance of different methods: peak signal-noise ration (PSNR) and structural similarity (SSIM)^5^ [21].

In the experiments, we assume that the pixel values are within the interval [0, 255]. The added salt&pepper type of impulse noise *η*_*I*_ can have a value of either 0 or 255. For Gaussian noise, the values are also uniformly distributed within the interval [0, 255]. For the parameters in Algorithm 1, we empirically set *λ*_1_ =0.9, *λ*_2_ =0.08, *λ*_3_ =0.08, and *β*_1_ = *β*_2_ = *β*_3_ = 200 for experiments. Note that we could tune the paramters to get better results, and we fix them in the experiments to illustrate the stability of the given method. For the parameters of “ASInpaint”, we keep the default settings of the provided code.

In Figure 2, we illustrate the visual performance of the two compared methods by four different simulated images with mixture noise (see Figure 2(a)) named “Lena”, “Cameraman”, “Phantom”, and “Satellite”. We added the Gaussian and impulse mixture noise on the images (see Figure 2(b)). In particular, we evaluate the effectiveness of the proposed method by the same image with different levels mixture noise (see Figure 2 the 1st and 3rd rows). Although the ASInpaint approach also obtained competitive results (see Figure 2(d)), the proposed method could obtain better visual performance, especially on the shape profile of the images (see Figure 2(e)). we have to emphasize that the visual performance of both methods seem to be not better than the recovered image by other literatures. The problem addressed is quite challenging that there are four unknown variables in the problem, such as the underlying clean image **X**, the mask **A**, the impulse noise **N**_**I**_, and the Gaussian noise **N**_**G**_. Although we may reduce to only two unknown variables **X** and **A**, it is still very difficult to recover the underlying clean image **X**. However, the given model has also recovered the relatively good visual results by the given algorithm.

The article "Blind Image Inpainting with Mixture Noise Using ℓ0 and Total Regularization" was published in 2022. Journal: Comput Math Methods Med.

Meanwhile, denoising results on a real color image by all competing methods (NLH method, NSNR method, WNNM method) is shown as Figure 3. The 15 test images used in image denoising experiments are shown as Figure 4. Inpainting results on images Starfish by different methods (Random mask with 75% missing values) are shown as Figure 5. Inpainting results on images Monarch by different methods (Text mask) are shown as Figure 6. These results show that PADMM algorithm has high performance of image denoising.

The quantitative comparisons of all methods are reported in Table 1, which indicates that the PADMM algorithm can improve the performance and yield the best quantitative results. Meanwhile, the paper tests the performance of NLH, KSVD, BM3D and WNNM algorithms on PSNR and SSIM of 15 pictures in the different value of *σ*_n_. The experimental results are shown in Tables 2 and 3. The results show that with the increase of *σ*_n_ value, the PSNR and SSIM of each picture gradually decrease, but the performance of these algorithms is significantly worse than PADMM algorithm.

## 5. Conclusions

In this paper, we present a novel optimization model and design the corresponding algorithm to address the challenging blind inpainting task with mixture noise. There are three main contributions in this work: 1) The model intetrates a *ℓ*_0_ sparse regularization to the binary mask, the total variation term to the underlying clean image and a *ℓ*_2_ regularization to describe the fidelity term; 2), Theproximal based alternating direction method of multipliers (PADMM) method was utilized and implemented to solve the optimization problem; 3) Experiments on some simulated examples with complex mixture noise are implemented, and the visual and quantitative results demonstrate the proposed method outperforms the other method.

## Figures and Tables

**Figure 1:** The flowchart of how to simulate the input image. Note that A and X are both blind and need to compute.

**Figure 2:** The visual comparisons between ASInpaint and the proposed method. (a) The ground-truth image; (b) The mask for the missing pixels; (c) The degraded image by Gaussian and impulse noise; (d) The recovered image by ASInpaint [6]; (e) The recovered image by the proposed method.

The article "Blind Image Inpainting with Mixture Noise Using ℓ0 and Total Regularization" was published in 2022. Journal: Comput Math Methods Med.

**Figure 3:** Denoising results on a real color image by all competing methods.

**Figure 4:** The 15 test images used in image denoising experiments.

**Figure 5:** Inpainting results on images Starfish by different methods (Random mask with 75% missing values).

**Figure 6:** Inpainting results on images Monarch by different methods (Text mask).

**Algorithm 1:** Solve the optimization model (5) by PADMM.

**Table 1:** The quantitative performance of Figure 2 for the two compared methods with the corresponding noise setting, i.e., missing proportion for impulse noise Ni and the *a* for Gaussian noise Ng.

Image	Noise setting	ASInpaint [6]		PADMM	
		PSNR	SSIM	PSNR	SSIM
Lena	50% missing *σ*_n_ = 15	21.82	0.6347	22.78	0.6650
Cameraman	30% missing *σ*_n_ = 19	19.13	0.5435	19.60	0.5630
Lena	10% missing *σ*_n_ = 15	24.29	0.7175	24.49	0.7240
Phantom	10% missing *σ*_n_ = 0.4	49.25	0.9657	49.35	0.9666
Satellite	10% missing *σ*_n_ = 15	22.41	0.6446	22.54	0.7662

**Table 2:** Denoising results (PSNR, SSIM) by competing methods on 15 test images.

	NLH		KSVD		BM3D		WNNM	
	PSNR	SSIM	PSNR	SSIM	PSNR	SSIM	PSNR	SSIM
*σ_n_* =15								
C.man	32.0054	0.9001	31.4074	0.8926	31.9152	0.9007	32.1768	0.9036
House	35.2832	0.8981	34.308	0.8758	34.9447	0.8907	35.1533	0.8909
Peppers	32.9416	0.9087	32.2062	0.8987	32.7017	0.9064	32.974	0.9098
Straws	28.5721	0.9285	28.3231	0.9262	28.5618	0.9317	29.1396	0.9396
Leaves	32.0951	0.9697	30.8806	0.9562	31.7233	0.9659	32.8266	0.9735
StarFish	31.4140	0.9007	30.7377	0.8931	31.1458	0.9007	31.8255	0.9081
Monarch	32.1065	0.9388	31.3864	0.9291	31.8597	0.9360	32.7178	0.9424
Airplane	31.4084	0.9025	30.7955	0.8937	31.0768	0.8995	31.4004	0.9029
Ma	31.9838	0.8657	31.4910	0.8544	31.9293	0.8667	32.123	0.8701
J.Bean	36.1662	0.9708	35.5188	0.9635	35.7038	0.9678	36.5642	0.9735
Couple	31.9414	0.8692	31.4498	0.8540	32.1087	0.8761	32.1818	0.8746
Parrot	31.3826	0.8919	31.0367	0.8915	31.3760	0.8944	31.6071	0.8968
Barbara	32.8384	0.9216	32.4214	0.9099	33.1141	0.9228	33.6114	0.9277
Boat	31.9944	0.8483	31.7033	.8410	32.1401	0.8534	32.2800	0.8549
Lena	34.1902	0.8953	33.7410	0.8851	34.2716	0.8950	34.3822	0.8973

*σ_n_* =30								
C.man	28.8607	0.8402	28.0158	0.8157	28.6377	0.8366	28.7827	0.8399
House	32.4570	0.8502	31.1754	0.8305	32.0871	0.8474	32.551	0.8523
Peppers	29.5743	0.8540	28.791	0.8407	29.2799	0.8500	29.4916	0.8567
Straws	24.4253	0.8038	24.3021	0.7964	24.8358	0.832	25.2457	0.8497
Leaves	28.1228	0.9333	26.9665	0.9118	27.8111	0.9275	28.6083	0.9389
StarFish	27.8924	0.8331	27.2325	0.8130	27.6535	0.8286	28.0689	0.8357
Monarch	28.7220	0.8891	28.0109	0.8717	28.3641	0.8817	28.9135	0.8926
Airplane	27.9736	0.8439	27.2595	0.8252	27.5592	0.8366	27.8176	0.8438
Ma	28.9999	0.7803	28.3244	0.7514	28.8597	0.7798	28.9798	0.7818
J.Bean	32.0428	0.9321	31.6162	0.9227	31.9669	0.9350	32.5005	0.9438
Couple	28.9726	0.7964	28.9726	0.7463	28.8691	0.7943	28.9679	0.7945
Parrot	28.3200	0.8319	27.5551	0.8186	28.1184	0.8313	28.3202	0.8346
Barbara	29.8374	0.8746	28.6006	0.8226	29.8136	0.8682	30.3086	0.8812
Boat	29.1663	0.7785	28.4093	0.7440	29.1172	0.7791	29.2262	0.7792
Lena	31.3194	0.8474	30.4192	0.8245	31.2621	0.8443	31.4315	0.8502

*σ_n_* =50								
C.man	26.3466	0.7903	25.7361	0.7451	26.1130	0.7822	26.4176	0.7848
House	30.5178	0.8306	27.9468	0.7602	29.6939	0.8116	30.3325	0.8231
Peppers	27.0524	0.8063	26.0368	0.7695	26.6834	0.7932	26.9123	0.8008
Straws	21.6929	0.6308	21.3263	0.5800	22.2874	0.6898	22.7261	0.7305
Leaves	25.3567	0.8907	24.2136	0.8571	24.6818	0.8677	25.4721	0.8925
StarFish	25.2100	0.7492	24.3876	0.7125	25.0443	0.7429	25.4327	0.7596
Monarch	26.2902	0.8354	25.1663	0.7937	25.8186	0.8196	26.3170	0.8350
Airplane	25.3611	0.7821	24.6200	0.7431	25.1022	0.7716	25.4244	0.7850
Ma	26.8762	0.7031	26.0308	0.6625	26.8081	0.7051	26.9373	0.7090
J.Bean	29.6937	0.9114	28.1745	0.8526	29.2595	0.8998	29.6351	0.9098
Couple	26.4604	0.7057	25.3037	0.6309	26.4638	0.7064	26.6436	0.7135
Parrot	25.9856	0.781	25.4187	0.7540	25.8984	0.7804	26.0926	0.7847
Barbara	27.4833	0.8128	25.5600	0.7191	27.2254	0.7942	27.7887	0.8199
Boat	26.8625	0.7032	25.9357	0.6569	26.7808	0.7050	26.9693	0.7083
Lena	29.2023	0.8069	27.8701	0.7606	29.0502	0.7989	29.2512	0.8059

*σ*_n_ =75								
C.man	24.7529	0.7492	23.1804	0.6550	24.3254	0.7334	24.5520	0.7353
House	28.5325	0.7963	25.3369	0.6800	27.5085	0.7640	28.2378	0.7887
Peppers	25.1632	0.7510	23.5163	0.6835	24.7341	0.7364	24.9152	0.7418
Straws	20.4422	0.5214	19.2792	0.3604	20.5588	0.5440	21.0039	0.6040
Leaves	23.0093	0.8306	20.7623	0.7296	22.4889	20.8070	23.0594	0.8350
StarFish	23.2220	0.6642	22.1093	0.6027	23.2746	0.6667	23.4720	0.6801
Monarch	24.4982	0.7831	22.9080	0.7183	23.9073	0.7553	24.3075	0.7754
Airplane	23.6914	0.7289	22.3293	0.6611	23.4749	0.7145	23.7407	0.7302
Ma	27.4366	0.8824	25.4310	0.7616	27.2153	0.8565	27.4233	0.8707
J.Bean	27.4366	0.8824	25.431	0.7616	27.2153	0.8565	27.4233	0.8707
Couple	24.9190	0.6422	23.5776	0.5511	24.6988	0.6257	24.8577	0.6369
Parrot	24.3794	0.7421	23.3786	0.6820	24.1856	0.7302	24.3698	0.7410
Barbara	25.6379	0.7430	23.0497	0.6032	25.1238	0.7108	25.8123	0.7486
Boat	25.3021	0.6487	23.9756	0.5795	25.1196	0.6407	25.2951	0.6465
Lena	27.5996	0.7706	25.7484	0.6939	27.2569	0.7510	27.5432	0.7657

*σ*_n_ =100								
C.man	23.5329	0.7050	21.6712	0.5762	23.0813	0.6922	23.3579	0.6968
House	26.7203	0.7589	23.6751	0.6186	25.8723	0.7196	26.6640	0.7536
Peppers	23.8028	0.7076	21.8289	0.6238	23.3946	0.6876	23.4485	0.6978
Straws	19.4043	0.4004	18.3801	0.2655	19.4303	0.4223	19.6878	0.4537
Leaves	21.5963	0.7844	18.2896	0.5934	20.9095	0.7481	21.5658	0.7884
StarFish	22.1677	0.6158	20.9669	0.5397	22.0977	0.6051	22.2263	0.6170
Monarch	23.1498	0.7322	20.5568	0.6154	22.5185	0.7017	22.9500	0.7257
Airplane	22.6891	0.6953	20.8416	0.5773	22.1094	0.6710	22.5529	0.6854
Ma	24.4735	.6139	23.3894	0.5482	24.2237	0.5975	24.3584	0.6048
J.Bean	26.1801	0.8561	23.6984	0.6911	25.8010	0.8175	26.0293	0.8337
Couple	23.7407	0.5835	22.6183	0.4992	23.5107	0.5661	23.5597	0.5702
Parrot	23.1367	0.7053	21.8362	0.6820	22.9593	0.6892	23.1863	0.7045
Barbara	24.4712	0.6960	21.8834	0.5332	23.6243	0.6426	24.1098	0.6862
Boat	24.2023	.6073	22.7806	0.5246	23.9703	0.5932	24.1098	0.5981
Lena	26.4509	0.7428	24.3508	0.6387	25.9548	0.7085	26.2127	0.7256

The article "Blind Image Inpainting with Mixture Noise Using ℓ0 and Total Regularization" was published in 2022. Journal: Comput Math Methods Med.

**Table 3:** The average PSNR & SSIM values by comprting methods on the 15 test images: The best results are highlighted in bold.

	*σ*_n_ =15		*σ*_n_ = 30		*σ*_n_ =50		*σ*_n_ =75		*σ*_n_ =100	
	PSNR	SSIM	PSNR	SSIM	PSNR	SSIM	PSNR	SSIM	PSNR	SSIM
BM3D	32.3048	0.9072	28.9490	0.8448	26.4607	0.7779	24.6126	0.7120	23.2972	0.6575
KSVD	31.8271	0.8977	28.3099	0.8223	25.5818	0.7332	23.2684	0.6372	21.7845	0.5685
NLH	32.4216	0.9073	28.3099	0.8459	26.6928	0.7826	24.9342	0.7269	23.4999	0.6747
WNNM	**32.7309**	**0.9116**	**29.2809**	**0.8517**	**26.8235**	**0.7908**	**24.9360**	**0.7300**	**23.6013**	**0.6761**

## Data Availability

The data that support the findings of this study are available from the corresponding author, [author initials], upon reasonable request.
